This article has been retracted.

# Serum Markers CA125, CA153, and CEA along with Inflammatory Cytokines in the Early Detection of Lung Cancer in High-Risk Populations

**DOI:** 10.1155/2022/1394042

**Published:** 2022-10-17

**Authors:** Guangping Li, Hongxin Zhang, Lei Zhang, Huaqun Liu, Songlin Li, Yanan Wang, Xiaoyun Deng

**Affiliations:** ^1^Department of Clinical Laboratory, Tangshan Gongren Hospital, No. 27, Wenhua Road, Lubei District, Tangshan City, Hebei Province, China; ^2^Department of Respiration, Tangshan Gongren Hospital, No. 27, Wenhua Road, Lubei District, Tangshan City, Hebei Province, China; ^3^Deportment of Oncology, Tangshan Gongren Hospital, No. 27, Wenhua Road, Lubei District, Tangshan City, Hebei Province, China

## Abstract

Lung cancer mortality and morbidity rates are the first among malignant tumors. It is extremely crucial to pay more attention to the early diagnosis and treatment of lung cancer and to grasp and judge the progress of the patient's condition promptly. In this study, lung cancer patients' early diagnosis with tumor markers and inflammatory variables is examined. The general surgery department of our hospital treated 98 patients with lung cancer and 100 patients with benign pulmonary hyperplasia from January 2017 to February 2018. Additionally, 100 healthy subjects who completed physical examinations during this time period were included. Based on the findings of the pathological examination, 100 patients with benign pulmonary hyperplasia were chosen as the benign group, 100 patients with lung cancer were chosen as the malignant group, and 100 healthy individuals were chosen as the healthy group. The tumor markers carbohydrate antigen 125 (CA125), CA153, and carcinoembryonic antigen (CEA), as well as inflammatory factors such as tumor necrosis factor- (TNF-) and high-sensitivity C-reactive protein, were measured in the venous blood of three groups of patients (hs-CRP). There was no discernible difference in tumor marker levels between the benign and healthy groups (*P* > 0.05). In comparison to the benign and healthy groups, the malignant group had higher serum levels of CA153, CA125, and CEA (*P* 0.05). Between the benign and healthy groups, there was no discernible difference in the levels of inflammatory factors (*P* > 0.05). TNF- and hs-CRP serum levels were observed to be higher in the malignant group compared to the benign and healthy groups (*P* 0.05). The combined detection of CA153 + CA125 + CEA + TNF − +hs − CRP showed the highest sensitivity and specificity, which were, respectively, 62.22 percent and 92.00 percent, when compared to single or mixed detection of tumor markers or inflammatory factors solely. Serum levels of inflammatory agents TNF- and hs-CRP may be related to the pathophysiology and other functions of patients with lung cancer, as well as to the development and metastasis of the disease. These markers include CA153, CA125, and CEA. For the early detection of lung cancer and the evaluation of the disease's severity, the detection of tumor markers in combination with inflammatory variables has a significant reference value.

## 1. Introduction

There has been significant progress in the diagnosis and therapy of lung cancer in the last ten years; however, the mortality rate of lung cancer still ranks first in the world. Lung cancers are allocated into two subtypes of histological classification: nonsmall cell lung cancer and small cell lung cancer (SCLC). As a malignant tumor with high lethality, the 5-year survival rate of lung cancer is only 4-17.7%. Radical resection with or without chemoradiotherapy is an effective treatment strategy for early-stage patients, including stages I, II, and a portion of stage III [1]. Unfortunately, because the early symptoms of lung cancer are insidious and the detection rate is low, most lung cancer patients are diagnosed at an advanced stage, which increases the difficulty of treatment and the risk of recurrence. Although molecular targeted therapy based on driver genes has gradually become the main force in the therapy of lung cancer, it has not fundamentally improved the high mortality rate of lung cancer, suggesting that the early diagnosis rate is a critical issue in improving the overall survival of lung cancer patients. In addition, there are many treatments for lung cancer, but the evaluation of cancer development and prognosis is limited owing to the tumor heterogeneity. Therefore, real-time monitoring of treating efficacy, quick, and precise recognition of drug resistance-related genes, the discovery of minimal residual disease, and the prognosis prediction are crucial to improve the therapeutic effect. At present, there are no clear measures for clinical diagnosis and treatment for lung cancer. In addition, the early symptoms are unknown, and most patients have missed the best treatment period when the disease is to be detected, resulting in continuous aggravation of the disease and missed treatment period. Tumor markers have the advantages of safety and noninvasiveness and have a certain guiding significance in cancer diagnosis. The early detection rate is low due to the lack of early signs. Most of them are in the middle and late stages when they are clinically diagnosed, and they lose the best chance of surgical treatment.

Therefore, early diagnosis and timely symptomatic treatment are the keys to improving the prognosis. In our study, we randomly choose a total of 98 patients with lung cancer and 100 patients with benign pulmonary hyperplasia from January 2017 to February 2018. We applied SPSS 20.0 to analyze data. We measured the tumor markers carbohydrate antigen 125 (CA125), CA153, and carcinoembryonic antigen (CEA), as well as inflammatory factors such as tumor necrosis factor- (TNF-), and high-sensitivity C-reactive protein and compared results between benign and healthy groups. With the deepening of serum tumor markers in clinical research, carbohydrate antigen 15-3 (CA 15-3), CA 125, and carcinoembryonic antigen (CEA), as markers associated with lung cancer, have significant advantages in the diagnosis of lung cancer.

## 2. Materials and Methods

### 2.1. Clinical Sample Collection

A total of 98 patients with lung cancer and 100 patients with benign pulmonary hyperplasia who were treated at the general surgery department of our hospital from January 2017 to February 2018 were randomly selected, and 100 healthy subjects who received physical examination during this period were included. From the results of the pathological analysis, 98 lung cancer patients were included in the malignant group, 100 patients with benign pulmonary hyperplasia were included in the innocent group, and 100 healthy subjects were selected as the healthy group. The mean age of patients in the malignant group was 42.06 ± 10.21 years, and that in the benign and healthy groups was 42.23 ± 10.41 and 42.15 ± 10.34 year, respectively. No statistical difference was found in the general data among the three groups of respondents (*P* > 0.05).

Inclusion criteria are (1) the pathological results meet the diagnostic criteria for lung cancer, (2) the first discovery of lung cancer, (3) unilateral lung cancer, and (4) sign the informed consent.

Exclusion criteria are (1) patients with a history of other malignant tumors, (2) pregnant or lactating women; (3) patients with inflammatory or metastatic lung cancer, (4) patients with cardiopulmonary insufficiency, and (5) the mentally ill.

### 2.2. Check Metrics

Fasting blood samples of subjects in the three groups were all collected in the morning, and 3 mL of venous blood was collected and centrifuged for use. (1) Tumor marker indicators: an automatic electrochemiluminescence immunoassay analyzer (Roche, model: RocheE601) was applied to detect serum CA125, CA153, and CEA levels. (2) Inflammatory factor indicators: an automatic immunoluminescence analyzer (Siemens, Germany, model: DPC IMMULTE2000) was applied to detect the level of tumor necrosis factor-*α* (TNF-*α*), and an automatic specific protein analyzer (Spain BIOSTEC company, model: BiosystemsA15) was used to detect the level of hs-CRP.

### 2.3. Statistical Methods

All data were analyzed by SPSS 20.0, and the general information of researchers, tumor markers, and inflammatory factors were expressed as (*x* − ±*s*) and analyzed by the *t* test. *P* < 0.05 was set to the cut-off threshold for statistical significance.

## 3. Experimental Results

### 3.1. Comparison of Tumor Marker Levels among Three Groups

The levels of tumor markers showed no significant difference between the benign and healthy groups (*P* > 0.05). However, the serum levels of CA153, CA125, and CEA were significantly higher in the malignant group than those in the benign and healthy groups (*P* < 0.05).  Table 1 shows the comparison of serum tumor marker levels in three groups of subjects.

### 3.2. Comparison of Inflammatory Factors among Three Groups

Serum levels of inflammatory factors presented no significant difference between the benign and healthy groups as well (*P* > 0.05), but significantly higher levels of TNF-*α* and hs-CRP were found in the malignant group (*P* < 0.05) (Tables 1 and 2).

### 3.3. Single and Combined Detection of Tumor Markers and Inflammatory Factors

Compared to detection of only tumor markers or inflammatory factors, combined detection of these biomarkers CA153 + CA125 + CEA + TNF − *α* + hs − CRP has the highest sensitivity and specificity, which were 62.22% and 92.00%, respectively, as shown in Table 3.

## 4. Discussion

Tumor markers are formed by the interaction of the tumor, tumor tissue, and the patient's body. They can be detected by examining the patient's blood, tumor tissue, and tissue fluid and can reflect the tumor growth in the patient's body to a certain extent. It is reported that the process of tumor formation is long and complex. The error of a single tumor marker in detecting lung cancer is high, and the types of tumor diseases that different tumor markers can reflect are also different. Therefore, the combined detection of multiple tumor markers can be used to improve the lung cancer-diagnosis rate. NSE is an enolase isoenzyme produced in malignant tumors of peripheral nervous tissue, neuroectoderm, and central nervous system. NSE has been demonstrated to have a certain guiding significance in the diagnosis of SCLC and has high sensitivity and specificity for the detection of SCLC CEA is produced in human embryonic tissue and is a nonorgan-specific tumor antigen, which can promote tumor metastasis to a certain extent. When healthy people have lung cancer, tumor cells can secrete a large amount of CEA and transfer it into the human blood circulatory system, resulting in a significant rise in the CEA level in the human body. Therefore, when diagnosing adenocarcinoma, the detection of CEA level has certain clinical guiding significance. CA125 is a glycoprotein complex and cannot enter the human blood circulatory system due to the influence of cell junctions and cell basement membranes in healthy humans. When human tumor cells are necrotic or lysed, the protease is stimulated and activated, leading to the degradation of keratin, and CYFR A21-1 will enter the human blood circulatory system. CYFR A21-1 belongs to the cytokeratin 19 fragment antigen, which is usually distributed in the monolayer of epithelial cells. When human tumor cells are necrotic or lysed, the protease is stimulated and activated, which leads to the degradation of keratin, and CYFR A21-1 will enter the in the human blood circulatory system. After testing, it can be observed that the lYFRA21-1 level is elevated. SCCA, as a serine protease inhibitor, is a typical squamous cell carcinoma-related protein. The protein can be expressed in normal squamous epithelium, pseudostratified columnar epithelium, and malignant tumor tissues derived from multistratified squamous epithelium. The results in Table 2 showed that the positive detection rates of serum tumor markers in patients with different types of lung cancer in the observation group were different, but the combined detection of five indicators has higher sensitivity and specificity than each single indicator (*P* < 0.05). It is further affirmed that the combined detection of multiple tumor markers in serum has a higher diagnostic accuracy.

## 5. Conclusion

To sum up, the protein has certain clinical diagnostic significance for various types of squamous cell carcinoma. According to the results of this paper, the serum levels of several tumor markers were noticeably higher in the malignant group than those in the benign and healthy groups (*P* < 0.05). Serum tumor marker levels were significantly increased. We believe that serum tumor markers have high clinical application value in diagnosing of lung cancer disease, but the effect of single tumor marker detection method is limited. However, we still have some limitations such as a limited sample size, which may influence the outcomes of our research. In the future, we need to collect more data and conduct more in-depth data analysis, which will improve the credibility of our conclusions.

## Figures and Tables

**Table 1:** Comparison of serum tumor marker levels in three groups of subjects.

Group	Number of cases	CA153 (U/mL)	CA125 (U/mL)	CEA (U/mL)
Malignant group	95	35.19 ± 17.03	21.51 ± 16.71	9.42 ± 4.29
Benign group	103	8.72 ± 4.02	13.09 ± 8.94	1.33 ± 1.63
Healthy group	106	8.22 ± 3.87	15.63 ± 9.52	1.09 ± 0.92
*F*		221.02	15.95	118.76
*P*		<0.001	<0.001	<0.001

**Table 2:** Comparison of serum inflammatory factor levels among three groups of subjects.

Group	Number of cases	TNF-alpha (pg/L)	hs-CRP (mg/L)
Malignant group	95	97.52 ± 16.39	16.85 ± 6.92
Benign group	103	79.25 ± 13.84	2.31 ± 1.09
Healthy group	106	68.33 ± 11.72	2.14 ± 1.18
*F*		101.97	263.81
*P*		<0.001	<0.001

**Table 3:** Single and combined detection of tumor markers and inflammatory factors.

Detection method	True positive	False positive	True negative	False negative	Sensitivity (%)	Specificity (%)
CA153 + CA125 + CEA	48	43	91	11	50.37	84.95
TNF − alpha + hs − CRP	39	45	81	15	43.29	82
CA153 + CA125 + CEA + TNF − alpha + hs − CRP	57	32	95	7	66.82	93.51

## Data Availability

All data is available upon reasonable requests.
